RETRACTED

# Downregulation of microRNA-15b-5p Targeting the Akt3-Mediated GSK-3*β*/*β*-Catenin Signaling Pathway Inhibits Cell Apoptosis in Parkinson's Disease

**DOI:** 10.1155/2021/8814862

**Published:** 2021-01-06

**Authors:** Jianzhong Zhu, Xue Xu, Yingyin Liang, Ronglan Zhu

**Affiliations:** ^1^Department of Neurology, Longmen County People's Hospital, Huizhou 516800, China; ^2^Department of Neurology, The First Affiliated Hospital of Sun Yatsen University, Guangzhou 510080, China

## Abstract

Parkinson's disease (PD) is an incurable progressive disorder resulting from neurodegeneration, and apoptosis is considered a dominant mechanism underlying the process of neurodegeneration. MicroRNAs (miRNAs), which are small and noncoding RNAs involved in many a biological process like apoptosis and regulation of gene expressions, have been found in postmortem brain samples of patients with PD, as well as *in vitro* and *in vivo* models of PD. To explore the impact of miR-15b-5p and Akt3 on apoptosis in the progression of PD, the method of quantitative reverse transcription polymerase chain reaction (qRT-PCR) was employed, and the analysis result showed upregulated expression of miR-15b-5p and downregulated expression of Akt3 in the serum of PD patients, MPP^+^-induced SH-SY5Y cells, and the brain tissues of MPTP-induced mice. Meanwhile, the dual-luciferase reporter assay was used to demonstrate the regulator-target interaction between miR-15b-5p and Akt3; flow cytometry and spectrophotometry revealed that transfection of miR-15b-5p mimic and si-Akt3 increased the rate of apoptosis and caspase-3 activity, whereas transfecting the miR-15b-5p inhibitor and Akt3-overexpression plasmid repressed the rate of apoptosis and caspase-3 activity in the MPP^+^-induced SH-SY5Y cell model and the MPTP-induced mouse model. Additionally, analysis of western blotting (WB) assays *in vivo* and *in vitro* revealed that proapoptosis proteins (Bax, caspase-3, GSK-3*β*, and *β*-catenin) showed markedly upregulated expression in the miR-15b-5p inhibitor and si-Akt3-overexpression groups, while the expression of an antiapoptosis gene (i.e., Bcl2) was downregulated. These analysis results indicate that downregulation of miR-15b-5p by targeting the Akt3-mediated GSK-3*β*/*β*-catenin signaling pathway would repress cell apoptosis in PD *in vivo* and *in vitro*. It is expected that the research findings would help find new therapeutic targets for treatment of PD.

## 1. Introduction

Parkinson's disease (PD), the most common neurodegenerative condition only second to the Alzheimer's, affects ~1% of individuals aged above 60 worldwide [1, 2]. One major pathological characteristic of PD is progressive and irreversible loss of the structure or function of dopaminergic neurons in the basal ganglia (the substantia nigra pars compacta region of the brain, in particular), which ultimately reduces the dopamine level to abnormal lows and leads to formation of Lewy bodies [3, 4]. As the dopaminergic neurons die, patients with PD progressively exhibit motor symptoms—resting tremor, muscular rigidity, bradykinesia, sympathetic instability, and the like—which severely degrade their quality of life [5]. Despite the rapid advancement in elemental research on the molecular mechanisms of PD pathogenesis over the past decades, systemic and effective treatment strategies for treating this disease are yet to be found [6, 7]. Recent studies have identified the presence of many dying neurons that exhibit chromatin condensation, DNA fragmentation, morphological changes, and engulfment of apoptotic bodies, in the dopaminergic neurons of autoptic brains of PD patients [8]. Moreover, many genes within the PD family (Parkin, HTRA2, PINK1, and DJ-1, for instance) were found to have played a role in regulating apoptosis by altering the biological functions of mitochondria [9, 10]. Therefore, these studies indicated that apoptosis, a selective process of cell deletion that requires specific cell death processes, may serve a critical role in PD progression and could be a novel target for therapies aimed at slowing or even stopping the disease progression [10].

RETRACTED

MicroRNAs (miRNAs), endogenous, single-strand noncoding, and highly conserved RNAs approximately 21-22 nucleotides in length, are found to play a regulatory role in the expression of approximately 30% of human genes. Specifically, they bind to the 3′-untranslated (3′-UTR) region of the target messenger RNA (mRNA), ultimately degrading the target mRNA and/or inhibiting its translation [11]. Presently, miRNAs are generally believed to be key regulators of the nervous system's functions, such as dendritic spine morphology, neurite outgrowth, synaptic plasticity, and neuronal differentiation. Therefore, disturbing the miRNA biogenesis pathways could potentially contribute to neurodevelopmental disorders and neurodegenerative diseases, including PD [12, 13]. For instance, miR-133b, a miRNA that has high expression in midbrain dopaminergic neurons and plays a regulatory role in the neurons' maturation and functions, is absent or at low levels in the substantia nigra of patients with PD [14]. Some other miRNAs like miR-7 and miR-153, in contrast, can bind directly to the *α*-synuclein (SNCA) mRNA directly and downregulate its expression. It should be noted that SNCA, which is primarily expressed in the neocortex, hippocampus, and substantia nigra, has been proved to be associated with the Lewy body pathology in PD [15]. Thus, in view of the effect of miRNAs on several endogenous genes, miRNA-based biomarkers may be considered to develop new strategies for the treatment of PD.

RETRACTED

The miR-15b-5p can induce cell apoptosis in human malignant tumors, such as hepatocellular carcinoma [16] and colorectal cancer [17]. A previous study also confirmed that miR-15b-5p in the plasma of patients with Alzheimer's could be used as a diagnostic biomarker [18], but the detailed role of this microRNA in the pathological process of PD remains to be explored. Additionally, inappropriate apoptosis control is the predominant mechanism that triggers the death of neurons and finally results in the pathogenesis of PD [8, 10]. Hence, in this study, we aim to explore whether miR-15-5p plays a role in the PD pathogenesis by regulating apoptosis in neurons and by regulating potential signaling pathways.

## 2. Materials and Methods

### 2.1. Ethics Statement and Specimen Collection

The present study has won approval and support from the Clinical Management Committee of Longmen County People's Hospital. Five healthy individuals and 10 patients who have been received a definite diagnosis with PD from at least three clinicians have signed the informed consent. Approximately 5 mL of fresh whole-blood specimen was collected from each subject, and the serum was immediately segregated within 1 h and stored at -80°C for subsequent qRT-PCR analysis. All experiments and analyses, including those involving human blood samples, were carried out as per the guidelines and regulations of the Clinical Management Committee of Longmen County People's Hospital.

### 2.2. Cell Culture

Samples of 293T cells and the human dopaminergic neuroblastoma SH-SY5Y cells obtained from American Type Culture Collection were cultivated in Dulbecco's modified eagle medium (Gibco, USA), supplemented with 10% fetal bovine serum (Gibco, USA), as well as L-glutamine (2 mmol/L), penicillin (100 U/mL), and streptomycin (100 *μ*g/mL) at 37°C in a humidified incubator containing 95% air and 5% CO_2_. For passaging, the SH-SY5Y cells, once reaching 80~90% confluence, were then treated with 0.25% trypsin (Sigma, USA).

### 2.3. qRT-PCR

To analyze the miR-15b-5p expression, a mirVana miRNA Isolation kit was employed to enrich the miRNA from clinical specimens and cell line samples. With the PrimeScript RT Reagent Kit (Takara Biotech, China) with miR-15b-5p-specific stem-loop primers, reverse transcription of the miRNA was performed by heating the samples at 16°C for 30 min and at 42°C for 40 min, followed by heat inactivation at 85°C for 5 min. The cDNA obtained thereby was amplified via qRT-PCR performed in an ABI PRISM® 7500 Sequence Detection System (Applied Biosystems, USA), featuring the following reaction conditions: reaction at 95°C for 2 min, 40 cycles of reaction steps (95°C for 15 s, 60°C for 32 s, and 95°C for 60 s), and 55°C for 30 s, followed by storage at 4°C. After each cycle, data were collected and used to generate a melting curve after the last step.

RETRACTED

The U6 snRNA and GAPDH served as the references for normalization of expression of miR-15b-5p and Akt3, respectively, and the relative gene expression was measured by employing the 2^−△△Ct^ method.  Table 1 lists the primers used in the qRT-PCR experiments.

### 2.4. Cell Counting Kit-8 Assay

To confirm the cytotoxic effect of 1-methyl-4-phenylpyridinium (MPP^+^) on SH-SY5Y cells, the Cell Counting Kit-8 (CCK8) (Dojindo, Japan) was used to measure cell viability first. MPP^+^ is a neurotoxin widely used to establish a neurotoxicity model in SH-SY5Y cells, and its effect resembles the neuron damages exhibited in PD. Briefly, 2 × 10^4^ cells/well was seeded in 96-well plates and treated with MPP^+^ of different concentrations (i.e., 0, 0.5, 1, 2, and 4 mM). 10 *μ*L CCK-8 reagent was added to each well at preset time points (0, 6, 12, 18, and 24 h from the start of cell culturing), and the mixture was incubated for an additional 2 h. Then, measurements of the optical density (OD) of cells in all wells, including the blank well without cells, were performed at an absorbance wavelength of 450 nm on a scanning microplate spectrophotometer (Thermo Fisher, USA). Each treatment group was composed of three independent wells.

### 2.5. Dual-Luciferase Reporter Assays

Prediction by the bioinformatics prediction of the TargetScan software indicated that there were two different binding sites between the 3′-UTR sequences in miR-15b-5p and Akt3. Therefore, the wild-type and mutant 3′-UTR sequences of Akt3 were synthesized (Sangon Biotech, Shanghai, China). Then, the sites between Xho I and Not I were used for cloning the fragments in the psi-CHECK2 basic luciferase reporter plasmid (Promega, USA). Cotransfection with these recombinant vectors was performed in 293T cells using Lipofectamine 2000 (Promega, USA).

### 2.6. Immunoblotting Detection

To further explore the roles that MPP^+^ plays in apoptosis of SH-SY5Y cells and primary neurons, the primary neurons from the substantial nigra were treated with MPP^+^, as described below. The insoluble material was removed after centrifugation at 12000 × g at 4°C for 10 min, before the total protein in the supernatant was determined by using the BCA protein assay kit (Beyotime, China). The protein was denatured, and then, 30 *μ*g of the protein was separated and loaded into wells on a 8 ~ 15% discontinuous SDS-PAGE gel. The result protein was then transferred to polyvinylidene difluoride membranes for 60 min using a 200 mA constant current. Thereafter, the membranes were sealed in 5% skimmed milk and the Tris buffer solution containing 0.1% Tween-20 (TBST) at room temperature for 2 h and cultured with primary antibodies against Akt3 (1 : 2000, Abcam, USA), Bcl2 (1 : 1000, Abcam, USA), Bax (1 : 1000, Abcam, USA), caspase-3 (1 : 500, Abcam, USA), GSK3*β* (1: 5000, Abcam, USA), *β*-catenin (1 : 5000, Abcam, USA), and GAPDH (1 : 10000, Abcam, USA) overnight at 4°C. Enhanced chemiluminescence reagents (Beyotime, China) were used to observe the immunoreactive bands. At last, the image processing software Image J was employed to compute the expression of related proteins.

RETRACTED

### 2.7. Flow Cytometry

The SH-SY5Y cells were incubated in 6-well plates at a density of 5 × 10^5^/cm^2^. When the cell density rose to 80%, the cells were transfected with the miR-15b-5p mimics, the miR-15b-5p inhibitor, the Akt3-overexpression plasmid, and the si-Akt3 plasmid. Then, 24 h after the transfection completed, the cells were treated with MPP^+^ (4 mM). The cells were harvested 24 h after different treatments for analysis of cell apoptosis, caspase-3 activity, and WB measurements. The harvested cells were first rinsed three times using cold phosphate-buffered saline (PBS) solution before being resuspended in the Annexin V binding buffer (Beyotime, China). Then, 10 *μ*L freshly prepared Annexin V-PI mixed reagent (Beyotime, China) was added to the cells for incubation at 25°C for 15 min without light. FACScan flow cytometry was used to analyze the samples within 30 min.

### 2.8. Examination of Caspase-3 Activity

The Caspase-3 Activity Kit (Beyotime, China) was used to measure the caspase-3 activity as per the manufacturer's instructions. Specifically, the harvested cells were centrifuged at 12000 × g for 10 min at 4°C; the majority of the supernatant after centrifugation was removed, while the cell precipitates were lysed using an ice-cold cell lysis buffer. The lysed cells were then mixed with the reaction buffer and 2 mM caspase-3 substrate to stay for 2 h at 37°C. Finally, the OD of the product cells was measured by spectrophotometry at 405 nm.

### 2.9. Animal Experiments

In the present study, five-week-old male C57BL/6 mice, weighing 15-18 g and provided by the Experimental Animal Center of Sun Yat-sen University, were used for animal experiments. The mice were raised in a standard pathogen free (SPF) environment at 25  ±  2°C under 12 h light-12 h darkness cycles. The mice were fed on autoclaved food and water throughout the study. All animal experiments in this work have won approval from the Animal Care and Use Committee of Sun Yat-sen University. The experiment mice were acclimated for at least 1 week before being randomly divided into four groups, with 9 mice per group. The four groups were a control group (intraperitoneally administrated a PBS solution only), a PD group, a PD + miR-15b-5p inhibitor group, and a PD + Akt3-overexpression group.

RETRACTED

The mice in the last two groups mentioned above (i.e., the PD + miR-15b-5p inhibitor group and the PD + Akt3-overexpression group) were pretreated with miR-15b-5p inhibitor and Akt3-overexpression plasmid, respectively, for 5 consecutive days. Next, 1-methyl-4-phenyl-1,2,3,6-tetrahydropyridine (MPTP, Sigma, USA) was freshly mixed with 0.9% saline and injected into mice in these two groups and those in the PD group intraperitoneally (i.p. 20 mg/kg) four times with an interval of 2 h. After 1 day, 3 days, and 7 days of MPTP treatment or PBS injections (the control group), the mice were euthanized by CO_2_ inhalation, and then, the brain tissues (which represent the whole brain homogenate) were dissected out for analyses of the expression of miR-15b-5p and Akt3, caspase-3 activity, and the expression of apoptosis-related proteins.

## 3. Results

### 3.1. miR-15b-5p and Akt3 Expressions Were Upregulated and Downregulated, Respectively, in the PD Group

To investigate the changes in miR-15b-5p and Akt3 expressions in PD patients, we employed qRT-PCR to quantify the expression of miR-15b-5p and Akt3 in healthy individuals and patients with PD. As the result reveals, PD patients showed much higher expression of miR-15b-5p (Figure 1(a)) but drastically lower expression of Akt3 (Figure 1(b)) than the healthy individuals in the control group. This suggested a potentially important role that aberrant expressions of miR-15b-5p and Akt3 might play in PD progression.

### 3.2. MPP^+^ Treatment Altered Cell Viability and the Expressions of miR-15b-5p and Akt3

A further probe into the role that miR-15b-5p and Akt3 play in PD progression was conducted by constructing a cell model of MPP^+^-induced neurotoxicity. The CCK8 assay revealed that the OD values representing cell viability declined gradually over time following treatment with MPP^+^ of different concentrations (Figure 2(a)). Moreover, the OD value reached the minimum after 24 h of treatment with 4 mM MPP^+^, and therefore, the treatment scheme of using MPP^+^ for 24 h was adopted in the following experiments. As Figures 2(b) and 2(c) show, the MPP^+^ group presented markedly higher expression of miR-15b-5p but considerably lower expression of Akt3 than the control group. The comparison indicates that the abnormal regulation of the miR-15b-5p and Akt3 expressions might exert a significant impact on progression of PD.

RETRACTED

### 3.3. miR-15b-5p Negatively Regulated Akt3

Analyses above suggested a negative correlation between miR-15b-5p expression and Akt3 expression. Hence, we assumed that miR-15b-5p might be directly targeting Akt3, and this assumption was supported by a bioinformatics analysis using the TargetScan software. Analysis based on the dual-luciferase reporter assays further revealed that the Renilla/Firefly luciferase activity altered in the mutant site 1 of the Akt3 3′-UTR but remained unchanged in the mutant site 2 (Figure 3(b)), which indicates that the mutant site 2 of Akt3 3′-UTR was the target binding site for miR-15b-5p. Besides, qRT-PCR and immunoblotting results showed the reduced Akt expressions (both mRNA and protein) in the miR-15b-5p treatment group but dramatically enhanced expression in the miR-15b-5p inhibitor group (Figures 3(c) and 3(d)). These findings further confirmed the interaction between miR-15b-5p and Akt3 at the molecular level.

### 3.4. Impact of miR-15b-5p and Akt3 on Apoptosis and the Apoptosis-Related Signaling Pathway *In Vitro*

In Figure 4(a) (in the left panel), cells of Annexin V^+^/PI^−^ resembled early apoptotic cells. Statistical analysis revealed that the MPP^+^, miR-15b-5p mimic, and si-Akt3 treatments induced apoptosis of SH-SY5Y cells, while the miR-15b-5p inhibitor and Akt3-overexpression treatments did not. Furthermore, the MPP^+^, miR-15b-5p, and si-Akt3 groups showed significantly higher caspase-3 activity than the control group; also, caspase-3 activity in the miR-15b-5p inhibitor and Akt3 groups was notably lower than that in the MPP^+^, miR-15b-5p, and si-Akt3 groups (Figure 4(b)). Compared with the expression levels of proapoptosis proteins (Bax, caspase-3, GSK-3*β*, and *β*-catenin) in the control group, those in the MPP^+^, miR-15b-5p, and si-Akt3 groups significantly increased but substantially decreased in miR-15b-5p inhibitor and Akt3 groups (Figure 4(c)). Meanwhile, the levels of the antiapoptosis protein (i.e., Bcl2) reduced notably in the MPP^+^, miR-15b-5p, and si-Akt3 groups but markedly elevated in the miR-15b-5p inhibitor and Akt3 groups (Figure 4(c)). Expression of these proteins presented a similar pattern in primary neurons in SH-SY5Y cells (Figure 4(d)). These findings indicated that miR-15b-5p might promote apoptosis by targeting Akt3 in an MPP^+^-induced PD cell model.

### 3.5. miR-15b-5p and Akt3 Expressions Increased and Decreased, Respectively, in the PD Mouse Model

The data on the clinical specimen and the MPP^+^-induced PD cell model verified possible involvement of miR-15b-5p and Akt3 in PD progression. Therefore, a PD mouse model was constructed to clarify their specific roles. It was observed that compared with the expression levels in the control group, the MPTP-induced PD mouse model showed higher miR-15b-5p expression and lower Akt3 expression than the control group (Figure 5). Also, the miR-15b-5p expression was significantly downregulated in the PD-miR-15b-5p inhibitor group, and the Akt3 expression was notably upregulated in the PD-Akt3-overexpression group, implying that the pretreatments with miR-15b-5p inhibitor and Akt3-overexpression plasmid were highly efficient.

RETRACTED

### 3.6. Impact of miR-15b-5p and Akt3 on Apoptosis and the Apoptosis-Related Signaling Pathway *In Vivo*

Caspase-3 activity was measured in the brain tissues of mice using the Caspase-3 Activity Kit. The measurement result reveals that caspase-3 activity in the PD group was substantially enhanced in comparison to the control group; though caspase-3 activity in the PD-miR-15b-5p inhibitor and the PD-Akt3-overexpression groups was also higher than in the control group, it was much lower than in the PD group (Figure 6(a)). Additionally, compared with the control group, the PD group showed markedly higher expression of proapoptosis proteins (Bax, caspase-3, GSK-3*β*, and *β*-catenin) and a much lower expression level of an antiapoptosis protein (Bcl2) (Figure 6(b)). The expression patterns of these proteins, however, reversed in the PD-miR-15b-5p inhibitor and the PD-Akt3-overexpression groups compared to the PD group (Figure 6(b)). Samples of these models at the Day 21th were chosen to examin the effect of prolonged exposure. The examination result reveals more pronounced impact of the treatment after 21 d (Figure 6(c)) than after 7 d (Figure 6(b)), despite the similar expression patterns. Taken together, these results clearly showed that suppression of miR-15b-5p might inhibit MPTP-induced apoptosis by regulating Akt3 *in vivo*.

## 4. Discussion

With the extension of life expectancy around the world, PD has gained increasing attention as a common neurodegenerative disorder [5]. Death of dopaminergic cells in the substantia nigra has been confirmed to bear close connection to the pathogenesis of PD, but the specific mechanism of neurodegeneration has yet to be elucidated [19, 20]. Accumulating evidence has revealed that miRNAs are negative regulators of target genes and play a role in such fundamental cell processes as development, differentiation, proliferation, survival, and apoptosis [21, 22]. Furthermore, most miRNAs have been found to play an essential role in PD pathology and development [23]. For instance, miR-155 regulates the SNCA-induced inflammatory responses in PD [24], and the serum level of miR-221 can serve as a biomarker for PD [25]. Moreover, in murine embryonic stem cell lines, mature miRNAs are eliminated by deleting Dicer (a type III ribonuclease required in the early stage of miRNA biosynthesis). Compared with wild-type embryonic stem cells, dopaminergic neuron phenotype is almost completely lost under appropriate differentiation signals, which may be due to increased cell apoptosis and reduced neurogenesis [14, 26]. Therefore, we intend to explore whether aberrantly expressed miRNAs in PD development play a role in death of dopaminergic neurons by regulating apoptosis-related genes or pathways. The present study found that miR-15-5p was significantly upregulated in patients with PD, the MPP^+^-induced SH-SY5Y cell model, and the MPTP-induced mouse model. Subsequently, Akt3, a serine/threonine protein kinase regulating cell survival and proliferation [27], was demonstrated to be notably downregulated in PD patients, the MPP^+^-induced SH-SY5Y cell model, and the MPTP-induced mouse model. Moreover, as revealed in Thome et al.'s study, microRNA-155 (miR-155) was significantly upregulated in an *in vivo* model of PD (developed using adeno-associated virus-mediated expression of alpha-synuclein); they also found that without miR-155, the mouse model experienced reduced proinflammatory responses to alpha-synuclein blocked alpha-synuclein-induced neurodegeneration. That is to say, miR-15b-5p may play a crucial role in the pathogenesis of PD via multiple mechanisms [24]. Located at 3q25.33 in humans, miR-15b-5p has been demonstrated to be a main cause of neural ischemic injuries [28, 29]. In addition, overexpression of miR-15b-5p has been proved to have a promoting effect on apoptosis of various cancerous cells [16, 17, 30]. For instance, it accelerates both endoplasmic reticulum stress and apoptosis by inhibiting Rab1A, which has been observed in human hepatocellular carcinoma *in vitro* and *in vivo* [31]. Moreover, activation of the Akt pathway is now considered a survival signal that enables cells to resist the stimulation of apoptosis [27]. For example, upregulated expression of periostin can activate the Akt signaling pathway through *α*v*β*3 integrins, improve the survival rate of cancer cells and endothelial cells, prevent stress-induced apoptosis, and significantly promote the metastatic growth of colon cancer [32]. In addition, the inverse expression patterns of miR-15b-5p and Akt3 suggest an interaction between miR-15b-5p and Akt3, which has been verified through dual-luciferase reporter assays. Then, the regulation of Akt3 after the overexpression and knockdown of miR-15b-5p was evaluated, and the results indicated that the miR-15b-5p mimic downregulated endogenous Akt3 (at both mRNA and protein levels) of 293T cells, while the miR-15b-5p inhibitor enabled upregulation, which further confirmed the regulator-target relationship between miR-15b-5p and Akt3. Thus, miR-15b-5p might play a proapoptosis role in the progression of PD by regulating Akt3.

RETRACTED

Apoptosis, a multistep process in mammalian cells, initially starts with the loss of mitochondrial integrity followed by the release of cytochrome *c*, which, combined with the apoptotic protease-activating factor (Apaf-1), activates the apoptosis signaling pathway (i.e., cysteine proteases, including caspase-3 and caspase-9), and ends up in cell death [33, 34]. In this work, an MPP^+^-induced SH-SY5Y cell model and an MPTP-induced mouse model were established to verify the roles of miR-15b-5p and Akt3 in apoptosis in the development of PD. In the cell model, the apoptosis rate and caspase-3 activity were remarkably higher in the miR-15b-5p and si-Akt3 groups than in the MPP^+^ group, whereas these indexes were markedly decreased in miR-15b-5p inhibitor and Akt3 groups when compared with miR-15b-5p and si-Akt3 groups. In the mouse model, caspase-3 activity in the PD-miR-15b-5p inhibitor and PD-Akt3-overexpression groups showed obviously lower caspase-3 activity than the PD group. In addition, the proteins of the apoptosis-related signaling pathway were examined by WB assays. During apoptosis, primary regulators include many Bcl-2 family members that contain antiapoptotic effectors (Bcl-2 and Bcl-xL, for instance) as well as their proapoptotic counterparts (Bad, Bid, Bik, Bax, and Bak) [35, 36]. Moreover, in response to the Akt signals, inactivation of GSK-3*β* by phosphorylation of the serine 9 residue (Ser9) triggers the stabilization, cytosolic accumulation, and *β*-catenin translocation, thus activating the expression of specific genes involved in the regulation of survival/apoptosis of different cells [37, 38]. For instance, palmitate has been proved to be able to induce apoptosis in cardiomyocytes by activating the Akt/GSK-3*β*-mediated *β*-catenin signaling pathway [39]. In this wok, we found that the blocking of miR-15b-5p and overexpression of Akt3 resulted in a dramatic decrease in Bax, caspase-3, GSK-3*β*, and *β*-catenin but a tangible increase in Bcl2 *in vivo* and *in vitro*, whereas overexpression of miR-15b-5p and inhibition of Akt3 led to a notable increase in Bax, caspase-3, GSK-3*β*, and *β*-catenin and a sharp drop in Bcl2 *in vitro*. Therefore, we have reason to conclude that miR-15b-5p might regulate apoptosis of neurons via the Akt3-mediated GSK-3*β*/*β*-catenin signaling pathway.

RETRACTED

Overall, we for the first time identified that miR-15b-5p and Akt3 were substantially increased and decreased, respectively, in PD both *in vivo* and *in vitro*. Moreover, we demonstrated a critical role of miR-15b-5p in apoptosis of neurons by regulating the Akt3-mediated GSK-3*β*/*β*-catenin signaling pathway (Figure 7). Hence, targeting the apoptosis-related Akt3/GSK-3*β*/*β*-catenin signaling pathway by miR-15b-5p could provide a novel therapeutic avenue for treating PD.

## Figures and Tables

**Figure 1:** miR-15b-5p and Akt3 expressions in serum samples of PD patients. (a) miR-15b-5p expression measured by qRT-PCR in healthy individuals and PD patients: miR-15b-5p was markedly upregulated in PD patients. (b) Akt3 mRNA expression measured by qRT-PCR in healthy individuals and PD patients: Akt3 was remarkably downregulated in PD patients ^∗^*P* < 0.05.

**Figure 2:** MPP^+^ treatment promoted the cytotoxic effect and changed miR-15b-5p and Akt3 expression in SH-SY5Y cells. (a) Neuronal viability monitored by CCK8 assays in SH-SY5Y cells was treated with MPP^+^ (0-4 mM) at specified time points. ^∗^*P* < 0.05. (b) Expression of miR-15b-5p under MPP^+^ treatment. ^∗^*P* < 0.05, ^∗∗^*P* < 0.01. (c) Expression of Akt3 under MPP^+^ treatment ^∗^*P* < 0.05.

**Figure 3:** Akt3 was proved a direct target of miR-15b-5p in regulation. (a) Binding site sequence comparisons between miR-15b-5p and the 3′-UTR sequence of Akt3. The complementary and mutated nucleotides were highlighted in red on the left panel. ^∗∗^*P* < 0.01. (b) Akt 3 expression in SH-SY5Y cells under treatments by the miR-15b-5p inhibitor or miR-15b-5p mimics. ^∗^*P* < 0.05. (c) The protein level of Akt3 in SH-SY5Y cells under treatments by miR-15b-5p inhibitor or miR-15b-5p mimics ^∗^*P* < 0.05.

**Figure 4:** miR-15b-5p-induced apoptosis by targeting Akt3 *in vitro*. (a) FACS plots of the apoptosis pattern in representative samples (left panel), corresponding statistical histogram in right panel. ^∗^*P* < 0.05, ^∗∗^*P* < 0.01. (b) Colorimetric assay of caspase-3 activity. miR-15b-5p enhanced the caspase-3 activity by regulating Akt3. ^∗^*P* < 0.05, ^∗∗^*P* < 0.01. (c) Immunoblotting (WB) analysis for apoptosis-related proteins in SH-SY5Y cells: miR-15b-5p promoted proapoptosis protein expressions via targeting Akt3. (d) WB analysis of apoptosis-related proteins in primary neurons: miR-15b-5p promoted proapoptosis protein expressions by targeting Akt3.

**Figure 5:** miR-15b-5p and Akt3 expressions in brain tissues of the PD mouse model. (a) miR-15b-5p expression quantified by qRT-PCR and normalized to GAPDH expression. ^∗^*P* < 0.05, ^∗∗^*P* < 0.01. (b) Akt3 expression tested by qRT-PCR and normalized to U6 snRNA expression, ^∗∗^*P* < 0.01.

RETRACTED

**Figure 6:** Suppression of miR-15b-5p inhibited MPTP-induced apoptosis by regulating Akt3 *in vivo*. (a) Colorimetric assay of caspase-3 activity: downregulating miR-15b-5p and upregulating Akt3 suppressed caspase-3 activity. ^∗^*P* < 0.05. (b) Protein expression of Bcl2, Bax, caspase-3, Akt, Gsk3*β*, and *β*-catenin in SH-SY5Y cells at 7 d after treatment to verify the role of miR-15b-5p and Akt3. Inhibition of miR-15b-5p and forced Akt3 attenuated expression of proapoptosis proteins. (c) Protein expression of Bcl2, Bax, caspase-3, Akt, Gsk3*β*, and *β*-catenin in SH-SY5Y cells at 21 d after treatment to verify the role of miR-15b-5p and Akt3. Inhibition of miR-15b-5p and forced Akt3 attenuated expression of proapoptosis proteins.

**Figure 7:** Working model of this study.

**Table 1:** Sequences of primers used for qRT-PCR assays.

miRNA or genes	Primer sequences
miR-15b-5p	(Reverse transcript primer): 5′-ACACTCCAGCTGGGTAGCAGCACATCATGGTT-3′ 5′-TGCATAGTCACAAAAG-3′ (sense) 5′-CTCAACTGGTGTCGTGGA-3′ (antisense)
U6 snRNA	(Reverse transcript primer): 5′-CTCAACTGGTGTCGTGGAGTCGGCAATTCAGTTGAGAAAAATATGG-3′ 5′-CTCGCTTCGGCAGCACA-3′ sense 5′-AACGCTTCACGAATTTGCGT-3′ antisense
Akt3 (human)	5′-GGGCGAGCTGTTTTTCCAT-3′ sense 5′-CGGTACACAATCTTTCCGGAAT-3′ antisense
GAPDH (human)	5′-AGAAGGCTGGGGCTCATTTG-3′ sense 5′-AGGGGCCATCCACAGTCTTC-3′ antisense
Akt3 (mouse)	5′-TGTCGCCAAAATCTATACACC-3′ sense 5′-ATTCCTTGCACATGGGTCA-3′ antisense
GAPDH (mouse)	5′-AGGCCGGTGCTGAGTATGTC-3′ sense 5′-TGCCTGCTTCACCACCTTCT-3′ antisense

## Data Availability

All data, models, and code generated or used during the study appear in the submitted article.
